The article "Electroadsorption Desalination with Carbon Nanotube/PAN-Based Carbon Fiber Felt Composites as Electrodes" was retracted in 2016. Reasons: plagiarized images; overlap with other authors' work; concerns about the citations.

# Electroadsorption Desalination with Carbon Nanotube/PAN-Based Carbon Fiber Felt Composites as Electrodes

**DOI:** 10.1155/2014/253713

**Published:** 2014-05-12

**Authors:** Yang Liu, Junbo Zhou

**Affiliations:** Engineering Research Center for Polymer Processing Equipment, Ministry of Education, College of Mechanical and Electrical Engineering, Beijing University of Chemical Technology, Beijing 100029, China

## Abstract

The chemical vapor deposition method is used to prepare CNT (carbon nanotube)/PCF (PAN-based carbon fiber felt) composite electrodes in this paper, with the surface morphology of CNT/PCF composites and electroadsorption desalination performance being studied. Results show such electrode materials with three-dimensional network nanostructures having a larger specific surface area and narrower micropore distribution, with a huge number of reactive groups covering the surface. Compared with PCF electrodes, CNT/PCF can allow for a higher adsorption and desorption rate but lower energy consumption; meanwhile, under the condition of the same voltage change, the CNT/PCF electrodes are provided with a better desalination effect. The study also found that the higher the original concentration of the solution, the greater the adsorption capacity and the lower the adsorption rate. At the same time, the higher the solution's pH, the better the desalting; the smaller the ions' radius, the greater the amount of adsorption.

## 1. Introduction

With economic development and population expansion, the scarcity of freshwater resources required for industrial and domestic use has been increasingly severe. Water purification has become a worldwide issue. Salt ions dissolved in water can be removed by distillation, reverse osmosis, electrodialysis, ion exchange, and so on. However, these methods have shortcomings such as high energy consumption, low water yield, or secondary pollution to the environment [1, 2]. In view of such problems, a new kind of water treatment method—electroadsorption desalination—has been developed recently. The mechanism is made so that a double layer can be formed between the electrode and solution in an electric field. Polar molecules or ions stored in the double layer can be removed; when electrodes become saturated, a reverse electric field can make the electrodes regenerate [3, 4]. Therefore, the choice of adsorbent materials and the molding process of electrode preparation are the keys to electroadsorption technology in practical applications. In order to be able to adsorb more charged particles, the adsorbent must possess a sufficiently large specific surface area, with porous carbon material being the best choice. This paper shall demonstrate how the chemical vapor deposition method was used to prepare CNT/PCF composite electrodes and then shall describe the process performed when studying electroadsorption desalination under different conditions.

## 2. Experiment

### 2.1. Materials and Instruments

Carbon nanotubes: Shenzhen Nanotech Port Co. (diameter: 40~60 nm; length: 0.5~500 *μ*m; purity: ≥95%); PAN-based carbon fiber felt: Shanghai Ai Ji Carbon Co., Ltd. (fixed carbon: >94%; sulfur content: <0.03%); LPCVD: Ideal Energy Equipment (Shanghai) Ltd.; 202-1 electrically heated drying oven; AP-2 HM conductivity meter: Xuzhou Ya Ming Appliances Co., Ltd.; DC power supply: 0–15 V, 0–2 A adjustable. BT00-100 M pump: Baoding Lan Ge Constant-Flow Pump Co., Ltd.; LEO-1530 SEM: Germany LEO Co., Ltd.

### 2.2. Pretreatment of Carbon Nanotubes and PAN-Based Carbon Fiber Felt

1. CNT pretreatment: put CNTs into 65% (mass fraction) HNO_3_ at 413 K for 4~5 hours, and have them neutralized, washed, and placed in centrifuge, after which CNTs with oxygen-containing reactive groups (such as –COOH and –OH) were obtained [5].
2. PCF pretreatment: put PAN-based carbon fiber felt into the HNO_3_ solution for 1 h, and then have it washed with distilled water to obtain neutralization and dried in vacuum at 393 K for 5 h [6].

### 2.3. CNT/PCF Electrode Preparation

The low pressure and low temperature thermal CVD system was adopted in this experiment, as shown in Figure 1. Ni was used as a catalyst and was deposited on the surface of graphite substrates. Hydrogen and acetylene were, respectively, used as the carrier gas and carbon feed stock, the flow rates of which were, respectively, controlled at 50 and 100 sccm. Reaction temperatures were at 823 K, and CNTs were dispersed on the PCF matrix. After deposition, the CNT/PCF composite had to be immersed into 1 mol/L HCl solution to remove the catalyst so that the influence of residues on electroadsorption could be avoided. The composite was then dried and shaped at 393 K to prepare for electrodes.

Electrode size in this electroadsorption experiment module is 100 mm × 50 mm × 2 mm (length × width × thickness). Assemble electrodes into desalinator, as shown in Figure 2. After being electrified, brine first flowed through this device at a certain rate, at which point the conductivity of the outlets could be tested, as shown in Figure 3.

## 3. Results and Discussion

### 3.1. Morphology Analysis of CNTs/PCF Composite

From Figures 4(a) and 4(b), we can see that carbon nanotubes wind around the PAN-based carbon fiber felt and form a three-dimensional conductive network nanostructure consisting of mesopores and a smaller amount of micropores. More micropores contact directly with the adsorbate, which can be exposed to the fiber surface for adsorption and desorption, meaning that the adsorption equilibrium can be reached quickly [7]. On the other hand, microspores shall increase the electrical double-layer overlapping effect and reduce electrosorption capacity according to the discussion led by Yang et al. [8]. Therefore, this kind of 3D network structure not only increases the external surface (the fiber diameter generally being between 10 and 13 *μ*m), but also suppresses the micropores' distribution as well. It thus becomes easier for micropores to contact with the adsorbate, so diffusion resistance decreases, which is beneficial for adsorptive separation without reducing the adsorption rate. Furthermore, since the nanotubes with curved winding structure are dispersed in the carbon felt, the resistivity of electrodes reduces while conductivity improves, with electrode strength also enhancing.

### 3.2. Impact of Adsorption Time on Electroadsorption Desalination

Prepare 1 mol/L NaCl solution, put 20 mL into electroadsorption module container, set closed-circuit voltage to 1.4 V, and adopt two kinds of electrodes (PCF electrode and CNT/PCF composite electrode) with the same mass. As shown in Figure 5, both desalination rates increase with the passage of time. When CNT/PCF composite electrodes are used, the conductivity of outlets decreases sharply within the first 20 minutes before then becoming gentle; after 80 minutes, this state remains generally unchanged. As for PCF electrodes, it takes a longer time to reach adsorption equilibrium. That is due to the increase in the mesopores' distribution, which reduces electroadsorption capacity and then accelerates the transfer of ions in the aperture, reducing energy consumption at the same time. With the comparison of the two kinds of electrodes, we can see that the outlet conductivity of CNT/PCF composite electrodes decreases more than that of PCF electrodes. According to the formula of electroadsorption capacitance (*C*) [9],

(1) $$\begin{array}{c} C=\int \frac{\varepsilon }{4\pi \delta }\cdot dS. \end{array}$$

This is true where *ε* is the effective permittivity of the electrical double layer, *δ* is the distance from the electrode surface to the center of the ion, which is equal to the thickness of the electric double layer, and *S* is the surface area of the electrode interface. The bigger the specific surface area of electrode aperture is, the greater the electroadsorption capacity becomes, and thereby the more obvious the desalination effect appears. The conclusion is that the desalination effect changes with the electrodes' specific surface area. Adding nanotubes increases the specific surface area of the electrode as analyzed above (1), allowing for the ability of electrode desalination to enhance indirectly.

### 3.3. The Impact of Closed-Circuit Voltage on Electroadsorption Desalination

Prepare 1 mol/L NaCl solution; put 20 mL into the container of electroadsorption module; set the closed-circuit voltage to 0.5 V, 0.8 V, 1.1 V, 1.4 V, 1.7 V, and 2 V and the adsorption time to 100 minutes; then test the conductivity of the outlets every 10 minutes. As shown in Figure 6, the adsorption capacity and rate increase with the raise in voltage. At 2 V, conductivity decreases at the fastest rate and has the minimum value, meaning that the higher the voltage, the better the effect of electroadsorption. The analysis shows that when the closed-circuit voltage increases, the electric double layer becomes thicker, and then the concentration of ions in the solution decreases more after a certain time. However, if the voltage is too high, solution electrolysis will appear, and energy consumption will increase [10]. With all these points considered, 1.4 V has been chosen as the ideal voltage.

### 3.4. The Impact of the Initial Concentration of Solution on Electroadsorption Desalination

Prepare 1 mol/L, 2 mol/L, 3 mol/L, 4 mol/L, and 5 mol/L NaCl solutions; put 20 mL into the electroadsorption module container, set the closed-circuit voltage to 1.4 V and adsorption time to 100 minutes, and adopt CNT/PCF composites as electrodes. The relationship of initial concentration of solution and desalination can be seen from Figure 7. It is obvious that the higher the initial concentration of solution is, the larger the adsorption capacity becomes at equilibrium. This is because the initial concentration determines the amount of ions in the solution. More ions have more chances to contact with electrode surfaces and can be easily adsorbed, with adsorption capacity being then able to enhance [11]. Yet, as the absolute increased number of ions in solution is far larger than the number of the adsorbed ones, the adsorption rate declines contrariwise, which means that the higher the initial concentration of NaCl solution is, the worse the adsorption effect becomes.

### 3.5. The Impact of Solution's pH Value on Electroadsorption Desalination

Set the pH value of solution to 6.13, 4.27, and 1.50. The adsorption capacity of CNT/PCF composite electrodes increases with the raise in the pH value while outlet conductivity decreases, as shown in Figure 8.

After pretreatment, a large number of reactive groups, like –COOH, phenolic hydroxyl (–OH), and so forth, have been formed on the surface of carbon nanotubes and PAN-based carbon fibers. These ions could be neutralized by NaOH and exchanged with cations [12–14]. Therefore, the more the reactive groups, the better the desalination effect.

### 3.6. The Removal of Different Ions

Prepare 1 mol/L CuCl_2_, CaCl_2_, and NaCl solutions. In the same adsorbing conditions (open-circuit voltage: 1.4 V; adsorption time: 100 minutes; used CNT/PCF composite electrodes), compare the removal effect of different cations. From Figure 9, one can see that, at the same voltage, the maximum adsorption capacity of CNT/PCF composite electrodes is Ca^2+^ > Cu^2+^ > Na^+^.

When applying voltage, ion adsorption works through electrostatic attraction (Coulomb force). The higher the ion's valence state, the bigger the electrostatic attraction between ions and electrodes. So, the adsorption rate of Ca^2+^ and Cu^2+^ is larger than that of Na^+^. For ions with the same valence state, electrostatic attractions between ions and electrodes are the same, and the electric adsorption effect may be decided by ionic radius. The smaller the ionic radius is, the easier the ions will move in the solution and the bigger the adsorption rate and adsorption capacity will be. As the radius of Cu^2+^ is bigger than the radius of Ca^2+^, the adsorption rate of Cu^2+^ is therefore larger than that of Ca^2+^.

## 4. Conclusions

1. The chemical vapor deposition method was used to prepare CNT (carbon nanotubes)/PCF (PAN-based carbon fiber felt) composite electrodes, which have a higher adsorption rate, lower energy consumption, and a better desalination effect. Such a 3D network structure has more surface area and narrower micropore distribution, which is beneficial for the adsorption and separation process as well as for electroadsorption.
2. The higher the initial concentration of solution, the larger the adsorption capacity and the lower the adsorption rate.
3. The acidic groups formed on the surface of carbon nanotubes and PAN-based carbon fibers result in the conclusion that the higher the pH of solution, the better the desalination effect. Electrostatic attraction between ions, electrodes, and ionic radius affects the adsorption of different ions. At the same voltage, the maximum adsorption capacity of CNT/PCF composite electrodes is Ca^2+^ > Cu^2+^ > Na^+^.

## Figures and Tables

**Figure 1:** LPCVD system.

**Figure 2:** Electroadsorption modules.

**Figure 3:** Electric adsorption desalination device.

**Figure 4:** (a) PCF electron microscopy scans and (b) electron microscopy scans of CNTs/PCF composite.

**Figure 5:** The adsorption time of CNT/PCF composite electrodes and PCF electrodes.

**Figure 6:** The outlets' conductivities at different voltages.

**Figure 7:** Adsorption capacity and desalination at different initial concentrations.

**Figure 8:** The outlets' conductivities at different pH values.

**Figure 9:** The outlets conductivity of different ions changed with time.

## References

[1] Wang YH, Chan KY, Li XY, So SK (2006). Electrochemical degradation of 4-chlorophenol at nickel-antimony doped tin oxide electrode. *Chemosphere*.

[2] Yasutoshi S, Kanako T, Mari Y, Kyosuke S (2012). Creation of carbon credits by water saving. *Water*.

[3] Han Y, Quan X, Chen S, Wang S, Zhang Y (2007). Electrochemical enhancement of adsorption capacity of activated carbon fibers and their surface physicochemical characterizations. *Electrochimica Acta*.

[4] Ryoo M-W, Seo G (2003). Improvement in capacitive deionization function of activated carbon cloth by titania modification. *Water Research*.

[5] Bottino A, Capannelli G, Comite A (2002). Preparation and characterization of novel porous PVDF-ZrO_2_ composite membranes. *Desalination*.

[6] Anderson MA, Cudero AL, Palma J (2010). Capacitive deionization as an electrochemical means of saving energy and delivering clean water. Comparison to present desalination practices: will it compete?. *Electrochimica Acta*.

[7] Xu P, Drewes JE, Heil D, Wang G (2008). Treatment of brackish produced water using carbon aerogel-based capacitive deionization technology. *Water Research*.

[8] Yang K-L, Ying T-Y, Yiacoumi S, Tsouris C, Vittoratos ES (2001). Electrosorption of ions from aqueous solutions by carbon aerogel: an electrical double-layer model. *Langmuir*.

[9] Wu HX, Zeng DY, Liu YM (2004). Inquiring into capital secondary sewage reuse for recycled cooling water in the thermal power plant. *Rurnal of the Central University for Nationalities (Natural Science Edition)*.

[10] Yang K-L, Yiacoumi S, Tsouris C (2003). Electrosorption capacitance of nanostructured carbon aerogel obtained by cyclic voltammetry. *Journal of Electroanalytical Chemistry*.

[11] Shen R, Andrews SA (2011). Demonstration of 20 pharmaceuticals and personal care products (PPCPs) as nitrosamine precursors during chloramine disinfection. *Water Research*.

[12] Liu Y, Zhou JB (2013). The study of modified pan-based carbon fiber felt as electrode in the electro-adsorption desalination. *International Journal of Electrochemical Science*.

[13] Tsuyoshi O, Ken M, Shoko T (2013). Synergistic water-treatment reactors using a TiO_2_-modified ti-mesh filter. *Water*.

[14] Shioyama H (2012). Carbon materials prepared by the use of metal-organic frameworks. *Carbon*.

